# Short-Axis PET Image Quality Improvement by Attention CycleGAN Using Total-Body PET

**DOI:** 10.1155/2022/4247023

**Published:** 2022-03-25

**Authors:** Chong Shang, Guohua Zhao, Yamei Li, Jianmin Yuan, Meiyun Wang, Yaping Wu, Yusong Lin

**Affiliations:** ^1^School of Information Engineering, Zhengzhou University, Zhengzhou 450001, China; ^2^Collaborative Innovation Center for Internet Healthcare, Zhengzhou University, Zhengzhou 450052, China; ^3^Central Research Institute, UIH Group, Shanghai 201807, China; ^4^Department of Medical Imaging, Henan Provincial People's Hospital, Zhengzhou 450003, China; ^5^School of Software, Zhengzhou University, Zhengzhou 450002, China; ^6^Hanwei IoT Institute, Zhengzhou University, Zhengzhou 450002, China

## Abstract

The quality of positron emission tomography (PET) imaging is positively correlated with scanner sensitivity, which is closely related to the axial field of view (FOV). Conventional short-axis PET scanners (200–350 mm FOV) reduce the imaging quality during fast scanning (2–3 minutes) due to the limitation of FOV, which reduce the reliability of diagnosis. To overcome hardware limitations and improve the image quality of short-axis PET scanners, we propose a supervised deep learning model, CycleAGAN, which is based on a cycle-consistent adversarial network (CycleGAN). We introduced the attention mechanism into the generator and focus on channel and spatial representative features and supervised learning using pairs of data to maintain the spatial consistency of the generated images with the ground truth. The imaging information of 386 patients from Henan Provincial People's Hospital was prospectively included as the dataset in this study. The training data come from the total-body PET scanner uEXPLORER. The proposed CycleAGAN is compared with traditional gray-level-based methods and learning-based methods. The results confirm that CycleAGAN achieved the best results on SSIM and NRMSE and achieved the closest distribution to ground truth in expert rating. The proposed method is not only able to improve the image quality of PET scanners with 320 mm FOV but also achieved good results on shorter FOV scanners. Patients and radiologists can benefit from the computer-aided diagnosis (CAD) system integrated with CycleAGAN.

## 1. Introduction

Positron emission tomography (PET), a widely used clinical imaging technique, can reflect metabolism in tissues by detecting the distribution of tracers in the human body. It is an effective means of current tumor detection [1] and early diagnosis [2] and offers advantages to the differentiation of benign and malignant tumors, and tumor staging and grading [3, 4]. PET image quality is a key factor affecting clinical diagnosis which is positively correlated with scanner sensitivity, and the sensitivity is closely related to the axial field of view (FOV). Large increases in signal collection efficiency can be realized by extending the FOV of the scanner [5]. Currently, clinically used PET devices mostly have an axial FOV of 200–350 mm and poor image quality in fast scanning. The uEXPLORER is the world's first total-body PET scanner, with a whole-body axial FOV (1940 mm) and ultrahigh sensitivity [6, 7]. The emergence of a total-body PET scanner with ultrahigh sensitivity can maximize the collection efficiency and provide high-quality images for PET image acquisition. However, currently, the cost of total-body PET is high (about five to six times that of a conventional scanner), and conventional short-axis PET scanner remains the mainstream device for PET image acquisition. How to improve the quality of PET image has been a focus in the nuclear medicine field [8].  Figure 1 shows the PET images of the brain, lungs, and abdomen. The images were obtained from the same person with short-axis PET TOF (320 mm FOV) and total-body PET uEXPLORER (1940 mm FOV) scanners in 5 minutes. The short-axis PET image had significantly lower quality than the total-body PET image in terms of noise and organ texture.

In clinics, the application of conventional short-axis PET scanner is limited by FOV. A single bed position scan enables the diagnosis of individual organs only, and the diagnosis of whole-body requires a combination of a series of serial scans obtained from many patient positions. A large amount of time-varying radiotracer distribution information can only be obtained from a part of the body at a time, and the whole-body PET images can be constructed through multiple serial scans within the specified time (15 minutes), with only 2–3 minutes per scan. Although this method can meet the needs of clinical diagnosis, it has the problems of significant image noise and unclear texture, which will reduce the reliability of diagnosis and offset the advantages of PET imaging.

Therefore, the purpose of our study is to improve the image quality of conventional short-axis PET scanners and further exert their clinical application value. The current research about how to technically enhance image quality mainly uses traditional and machine learning methods. Traditional methods are mainly used to resolve problems, such as low contrast, uneven intensity distribution, and edge blur of medical images. Machine learning methods learn the nonlinear mapping of low-quality PET (LQPET) and high-quality PET (HQPET) images, which are used as models for image quality enhancement.

Traditional image enhancement methods depend on image gray value distribution, which can be divided into frequency and spatial domain methods according to enhancement process space. Nonlocal means (NLM) [9] is a typical spatial method, which estimates the center point of the reference block by weighted averaging the self-similar image blocks in the image, so as to reduce the noise, but NLM does not protect the structure information of the original image enough. Dabov et al. [10] proposed block-matching and 3D filtering (BM3D) according to the similarity between image blocks. This method has a high signal-to-noise ratio, but the block operation will lead to fuzzy output and relatively high time complexity. Recently, these nonlearning-based methods have reached a bottleneck, whereas deep learning has made breakthroughs in medical image processing [2, 11–13]. The powerful mapping ability of deep learning brings a new idea to image enhancement. The introduction of the generative adversarial network (GAN) [14] in 2014 has provided new directions for many image research tasks. It has been used in medical image denoising, data simulation, classification, segmentation, and reconstruction [15–22] and in MRI, CT, PET, and other multimodal medical images. GANs can simulate data distribution, generate realistic images, and can solve the problem of the weak generalization ability of early generation models [23]. One of the original purposes of GAN is image enhancement, and their use in image enhancement has unique advantages. Ouyang et al. [24] used a GAN with texture feature matching and task-specific perceptual loss to generate standard-dose PET images from ultralow-dose PET images. Isola et al. [25] proposed the Pix2Pix supervised image-to-image translation framework, which is based on conditional generative adversarial network (CGAN) and uses a set of pairs and aligned images to train and learn the mapping between two image domains. To solve the problem of data mismatch, Zhu et al. [26] proposed the unsupervised training model of CycleGAN in 2017. This model can operate between the source domain *X* and target domain *Y* without establishing the one-to-one mapping of training data. Zhao et al. [27] proposed a nonlinear end-to-end mapping model S-CycleGAN to restore low-dose PET images of the brain. Zhou et al. [28] proposed the supervised deep learning model CycleWGAN, which was based on CycleGAN, to improve the quality of the low-dose PET images of the lungs and introduced Wasserstein distance into the loss function [29, 30]. The method achieved considerable results in preserving edges and SUV values. Inspired by these studies, we believe that an image postprocessing method based on deep learning can overcome the limitations of hardware and effectively improve the image quality of conventional PET device.

The attention mechanism was first proposed in the field of vision. Since the publication of Google Mind in 2014 [31], the attention mechanism has become popular. In this paper, an RNN model with the attention mechanism was used for image classification. Since the application of the attention mechanism in the field of natural language is processed by Bahdanau et al. [32], it has been applied to various fields and became a widely used technology. By connecting different modules in a weighted way, the attention mechanism allows the neural network to focus on relevant information rather than on irrelevant information. Vaswani et al. [33] proposed a machine translation model using the attention mechanism only, completely abandoning network structures, such as CNN and RNN, and achieved good results. Woo et al. [34] proposed a lightweight attention module and convolutional block attention module (CBAM), which can pay attention to channels and spatial dimensions and can be added to all conventional convolution layers. Woo et al. [34] tested the performance and versatility of CBAM in the ResNet network and visualized the results for improved interpretation. The attention–GAN framework proposed by Chen et al. [35] can learn accurate attention to improve image quality and can effectively prevent object deformation.

This paper proposes an image quality enhancement method named CycleAGAN, which can combine a cycle-consistent adversarial network (CycleGAN) [26] with the attention mechanism. The method was used in reconstructing HQPET images with low noise and fine texture on a short-axis PET device. Our main contributions are threefold:

1. For the reconstruction of realistic texture details, the attention mechanism module [34] is incorporated into the two generator networks of CycleGAN, which focus on channel and spatial representative features.
2. For the reduction of the dependence on the position information of the reference image and influence of deformation on the generated image, the images of the two image domains are aligned in space. The learning method of the network is changed to supervised learning, and supervised learning loss is added to the loss function to learn a nonlinear mapping that contains structural information.
3. To meet the amount of data required for deep learning, the sample size of the data set used in this experiment far exceeds the sample sizes of previous studies. In the training process, the image is input into the network in the form of a whole, and the global characteristics of the image can be learned. A large number of experiments are performed on images with different FOV to verify the effectiveness of the method.

## 2. Methods

The architecture of our proposed model, CycleAGAN, is shown in Figure 2. The network is a circular network composed of two mirrored GANs, including two generators (*G*_*AB*_, *G*_*BA*_) and two discriminators (*D*_*A*_, *D*_*B*_). *G*_*AB*_ represents the mapping from LQPET domain (*A*) to HQPET domain (*B*), and *G*_*BA*_ represents opposite mapping. In addition, the two discriminators *D*_*A*_ and *D*_*B*_ are designed to identify whether the output of each generator is real or fake. We trained the generators and discriminators simultaneously.

Quality from the LQPET image domain *A* to HQPET image domain *B* can be improved by training the generators *G*_*AB*_ and *G*_*BA*_. That is, we need to learn a mapping *G*_*AB*_ : *A*⟶*B* in order that the generated sample $\hat{b}=G_{AB}\left(a\right)$ is consistent with the distribution of the HQPET image domain *B*. Another reverse mapping of *G*_*BA*_ : *B*⟶*A* is added to make $\tilde{a}=G_{BA}\left(G_{AB}\left(a\right)\right)$ consistent with the LQPET image domain of *A* distribution and ensure cycle consistency, *G*_*BA*_(*G*_*AB*_(*a*)) ≈ *a*. To distinguish between the image generated by *A* and the real image in *B*, discriminator *D*_B_ was used to determine the category of the images. As the number of train epoch increases, *G*_*AB*_ and *D*_*B*_ are updated until the output result of *D*_*B*_ stabilizes to 0.5. In this case, the generated sample $\hat{b}$ is considered infinitely close to the HQPET image domain *B*. Similarly, the  *G*_*BA*_ and *D*_*A*_ training processes are the same as *G*_*AB*_ and *D*_*B*_.

### 2.1. Attention Module

The general structure of CBAM [34] includes two submodules: channel attention module and spatial attention module, as shown in Figure 3. In an intermediate feature map, the attention weight is deduced along the channel and spatial dimensions and then multiplied with the original feature map for feature adjustment.  Figure 4 shows the specific structures of the two submodules. *A* 1D channel attention map (*F*_*C*_) and a 2D spatial attention map (*F*_*S*_) are generated by the feature map through the channel and the spatial attention modules, respectively.

Channel attention can generate a channel attention feature map by using the channel relationship of features and can focus on the most valuable part of input features. In the calculation of channel attention, the spatial dimension of the input feature map needs to be compressed, and average pooling and maximum pooling are used simultaneously. This method not only facilitates the collection of unique texture features but also retains background information. After passing through the same convolution network, the average pooling and maximum pooling features are combined through element-wise summation and then activated by sigmoid for the acquisition of the channel attention *F*_*C*_.

Spatial attention uses the spatial relationship of features to generate a spatial attention feature map, focusing on the most informative part, which is a supplement to channel attention. In the computation of spatial attention, average pooling and maximum pooling are applied along the channel axis, and then, the results are concatenated into a valid feature descriptor. Then, the convolutional layer is used to generate spatial attention *F*_*S*_, which encodes the positions to be concerned or suppressed.

### 2.2. Generator Network

The network architecture of generators *G*_*AB*_ and *G*_*BA*_ is shown in Figure 5. The PET image is a single channel gray image, and the number of the input and output channels of the network is set to 1. ResNet is used as the basic network, and CBAM is introduced to make the network pay attention to subtle features and adjust the weights of the channel and spatial features. Change in the network structure of ResNet [36] is prevented by adding CBAM after the first layer convolution and before the last layer convolution successively.

The entire network comprises six convolutional layers, two CBAMs, and nine residue learning modules. The first convolution layer uses 64 sets of 7 × 7 convolution kernels to produce 64 channel feature maps and inputs them into CBAM and then through the two layers of the 3 × 3 down-sampling convolution, batch normalization, and ReLU layers. Nine sets of residual blocks are obtained, and each block contains two 3 × 3 convolution, batch normalization layers. The first is connected with ReLU, and the other is connected with bypass and ReLU. Reflection padding is used to reduce artifacts. Residual blocks are followed by two 3 × 3 up-sampling convolution, batch normalization, and ReLU layers. Then, the features are input into CBAM. Finally, a 7 × 7 convolution kernel and a tanh layer are used in estimating the HQPET image.

### 2.3. Discriminator Network

As shown in Figure 6, the discriminator has four 2D 4 × 4 CNN layers and a fully connected layer. Each CNN layer is followed by batch normalization and LeakyReLU layers as the activation function. Let *CkS*_*s − n*_ denote a convolution layer with a kernel size of *k* × *k*, a stride of *s*, *n* output channels, batch normalization, and LeakyReLU activation function with a slope of 0.2. The discriminator network architecture is as follows: C4S2-64, C4S2-128, C4S2-256, C4S1-512. After the last layer is obtained, we use convolution to produce a 1D prediction map output.

### 2.4. Loss Functions

The basic CycleGAN contains three kinds of losses: adversarial loss (ℒ_adv_), cycle-consistency loss (ℒ_cyc_), and identity loss (ℒ_id_). Although the CycleGAN was originally proposed to solve unsupervised learning model for unmatched data, the spatial consistency of images is still obtained through registration or reconstruction for the maintenance of quantized pixel values, the elimination of unnecessary differences between two image domains, and shifting of focus to the mapping of texture details. We add a supervised learning loss (ℒ_sup_) into the loss function. The total loss function is defined as

(1) $$\begin{array}{c} L=L_{\text{adv}}+\lambda_{c}L_{\text{cyc}}+\lambda_{i}L_{\text{id}}+\lambda_{s}L_{\text{sup}}, \end{array}$$

where *λ*_*c*_, *λ*_*i*_, and *λ*_*s*_ are hyperparameters.

Adversarial loss (ℒ_adv_) makes the PET image distribution generated by the generator close to the HQPET image distribution, including two parts defined in a similar way. One part is ℒ(*G*_*AB*_, *D*_*B*_) between *G*_*AB*_ and *D*_*A*_, and the other part is ℒ(*G*_*BA*_, *D*_*A*_) between *G*_*BA*_ and *D*_*A*_. The definition of adversarial loss is as follows:

(2) $$\begin{array}{c} {ℒ}_{adv}=\frac{1}{2}\left(ℒ\left(G_{AB},D_{B}\right)+ℒ\left(G_{BA},D_{A}\right)\right), \end{array}$$

where

(3) $$\begin{array}{c} \underset{G_{AB}}{\min}\underset{D_{B}}{\max}ℒ\left(G_{AB},D_{B}\right)=\\ -E_{x_{B}∼P_{B}}\left[D_{B}\left(x_{B}\right)\right]+E_{x_{A}∼P_{A}}\left[D_{B}\left(G_{AB}\left(x_{A}\right)\right)\right]+\lambda E_{\tilde{y}}\left[{\left({\left\|\nabla_{\tilde{y}}D_{B}\left(\tilde{y}\right)\right\|}_{2}-1\right)}^{2}\right]\;. \end{array}$$

Meanwhile, ℒ(*G*_*BA*_, *D*_*A*_) is defined in the same way as ℒ(*G*_*AB*_, *D*_*B*_).

Adversarial loss can only ensure that the generated PET and HQPET images have the same distribution. Cycle consistency loss can make *G*_*AB*_ and *G*_*BA*_ retain LQPET information and the consistency of content in the generation process. Thus, the generated PET image has high quality without change in its original image structure. Cycle consistency loss is defined as follows:

(4) $$\begin{array}{c} {ℒ}_{cyc}\left(G_{AB},G_{BA}\right)=E_{x_{A}∼P_{A}}\left[{\left\|G_{BA}\left(G_{AB}\left(x_{A}\right)\right)-x_{A}\right\|}_{1}\right]+E_{x_{B}∼P_{B}}\left[{\left\|G_{AB}\left(G_{BA}\left(x_{B}\right)\right)-x_{B}\right\|}_{1}\right]. \end{array}$$

In clinical applications, the input of *G*_*AB*_ may be HQPET. To ensure that *G*_*AB*_ can still output high-quality PET images, we define the identity loss as follows to enable the generator to achieve identity mapping and vice versa.

(5) $$\begin{array}{c} {ℒ}_{i\;d}\left(G_{AB},G_{BA}\right)=E_{x_{A}∼P_{A}}\left[{\left\|G_{BA}\left(x_{A}\right)-x_{A}\right\|}_{1}\right]+E_{x_{B}∼P_{B}}\left[{\left\|G_{AB}\left(x_{B}\right)-x_{B}\right\|}_{1}\right]. \end{array}$$

In this experiment, we use paired data and supervision loss is defined as follows:

(6) $$\begin{array}{c} {ℒ}_{\sup}\left(G_{AB},G_{BA}\right)=E_{x_{A}∼P_{A}}\left[{\left\|G_{AB}\left(x_{A}\right)-x_{B}\right\|}_{1}\right]+E_{x_{B}∼P_{B}}\left[{\left\|G_{BA}\left(x_{B}\right)-x_{A}\right\|}_{1}\right]. \end{array}$$

## 3. Experiments

### 3.1. Dataset

The experimental data came from the imaging department of Henan Provincial People's Hospital. All the data were collected using UNITED IMAGING total-body PET/CT uEXPLORER with 0.11 mCi/kg 18F-FDG. Data collection was started 45–60 minutes after injection, and the collection time is 5 minutes. A total of 386 age-matched patients (18–70 years old) were enrolled. The institutional ethics committee approved this study, and all participants gave informed written consent.

Given that the raw data collected by uEXPLORER come from the whole body of a patient, and the raw data collected was reconstructed into three consecutive bed positions. Each bed is 320 mm in length, and the beds correspond to the head (bed1), lung (bed2), and abdomen (bed3). To maximize the consistency between the estimated image and the LQPET image structure, uEXPLORER was used in reconstructing LQPET and HQPET with different reconstruction parameters. In each bed scan, the HQPET image is reconstructed with the signal from the full detector range (1940 mm), whereas the LQPET image was reconstructed with the signal from 320 mm FOV only [37]. The reconstruction algorithm was standard ordered-subset expectation maximization (OSEM) with time-of-flight (TOF). All necessary corrections such as scatter, normalization, dead time, random, attenuation, decay corrections were applied. The reconstruction parameters of bed1 are 300 mm visual field, 1.4 mm layer thickness, 4 iterations, 20 subsets; the reconstruction parameters of bed2 and bed3 are 500 mm visual field, 2 mm layer thickness, 2 iterations, 20 subsets. The difference between HQPET and LQPET reconstructed images lies in attenuation correction: the attenuation correction sequence used by HQPET comes from the whole detector range, while the attenuation correction sequence used by LQPET comes from the corresponding area of each bed. The image size of the bed1 was 150 × 150 × 230 with a voxel size 2 × 2 × 1.4 mm^3^, and the image size of the bed2 and bed3 was 192 × 192 × 160 with a voxel size 2.6 × 2.6 × 2 mm^3^. This procedure not only ensured the spatial consistency of the image but also enabled paired data to be trained with supervision. After verification, the image quality was equivalent when the reconstruction parameters on uEXPLORER were the same as those in the short-axis scanner.

After comparison and screening, the cases available for each bed composed of 344 head cases, with a total of 79,046 pairs of images; 361 cases of lung, with a total of 57,900 pairs of images; and 351 cases of abdomen, with a total of 56,746 pairs of images. Each bed position is trained separately, and the above data are randomly divided into training and test sets in an allocation ratio of 9 : 1. All PET voxel values are scaled to [−1,1] aiding to network training.

### 3.2. Experimental Settings

In the training process, we use an Adam [38] optimizer to minimize the total loss function (1) of CycleAGAN. The optimizer parameter is *β*_1_ = 0.5, *β*_2_ = 0.999. In the total loss function, the hyperparameters *λ*_*c*_, *λ*_*i*_, and *λ*_*s*_ are set at 10, 0.5, and 0.5, respectively, and *λ*_*s*_ is determined by experiment. The whole training epoch is set at 200, and the batch size is set at 32. In the first 100 epochs, the learning rate is set at 2*e* − 4. In the last 100 epochs, the learning rate is gradually reduced to 0. All implementation processes are performed using Python 3.6 and PyTorch 1.6 on PyCharm. All the experiments are performed on a Windows workstation with an Intel Xeon W-2135 64 GB CPU and two NVIDIA Quadro P5000 16 GB GPUs. With the current hardware facilities, model training for each bed is completed for 480 hours. Although the training requires a large amount of training time, it can result in good generalization performance because of the large amount of data. All the test images are entered in the model sequentially, and each image slice is generated for 9.4 milliseconds in average.

### 3.3. Evaluation Method

Image quality is analyzed according to radiologist rating and qualitative and quantitative data [39, 40].

Two radiologists with 10 years of experience assess image quality through blind review. The evaluation process has three aspects: overall impression, image noise, and focus significance. The doctor formulates a five-point scoring system based on three factors. The evaluation scale is shown in Table 1. The score is only used for images and does not consider other clinical data. First, the images to be evaluated are imported into the AMIDE software and then ranked by doctors in random for the reduction of deviation. Finally, the evaluation results of the two radiologists are sorted out for the consistency of image evaluation.

NRMSE, PSNR, and SSIM [41] are used in measuring the difference between the estimated PET image and ground truth HQPET image, and the performance of the proposed network model is quantitatively evaluated. The indicators are defined as follows:

(7) $$\begin{array}{c} \text{NRMSE}=\sqrt{\frac{\sum_{i=1}^{N}\sum_{j=1}^{M}{\left(x_{\text{ij}}-y_{\text{ij}}\right)}^{2}}{\sum_{i=1}^{N}\sum_{j=1}^{M}y_{\text{ij}}^{2}}}\times 100,\\ \text{PSNR}=20\times \log_{10}\left(\frac{\text{MAX}}{\sqrt{\text{MSE}}}\right),\\ \text{SSIM}=\frac{2\mu_{x}\mu_{y}+C_{1}}{\mu_{x}^{2}+\mu_{y}^{2}+C_{1}}\times \frac{2\sigma_{\text{xy}}+C_{2}}{\sigma_{x}^{2}+\sigma_{y}^{2}+C_{2}}, \end{array}$$

where *C*_1_ and *C*_2_ are constants;  *μ*_*x*_,  *μ*_*y*_,  *σ*_*x*_,  *σ*_*y*_, and *σ*_xy_ are the average and standard deviation of the plane centered on the pixel (*i*, *j*); MAX is the peak intensity of the image; and MSE is the absolute mean square error.

PSNR is the most widely used objective image evaluation index, which is based on the error between corresponding pixels. However, it does not consider the visual recognition and perception characteristics of human eyes, and the evaluation results are often different from people's subjective feelings [42]. The ratio between useful information and noise and image quality increases with PSNR. The SSIM value range is [0,1]. Image distortion decreases with increasing SSIM value. When the SSIM value is 1, the two images are the same.

## 4. Results

### 4.1. Result of Image Quality Improvement Experiments

The experimental results are obtained from 105 samples (34 in bed1, 36 in bed2, and 35 in bed3) in the test set. The proposed CycleAGAN method is compared with the original CycleGAN and Pix2Pix, NLM, and BM3D algorithms. CycleAGAN, CycleGAN, and Pix2Pix are deep learning methods, whereas NLM and BM3D are traditional image denoising methods. The filtering strength of NLM is set to 20, the hard thresholding of BM3D is set to 2.7, and the block size is 4. The HQPET images estimated by these methods are analyzed through qualitative and quantitative analyses and on the basis of radiologist rating.

#### 4.1.1. Qualitative and Quantitative Analysis

In qualitative analysis, representative sample images are selected from different beds. The three subgraphs in Figure 7 show the LQPET, HQPET, and generated HQPET sample images of representative subjects in the test set in three beds. The images are estimated with the five image quality improvement methods. Rows 1, 2, and 3 in each subgraph are PET images in the axial, coronal, and sagittal directions, respectively. In the first two columns of each subgraph, the quality of the LQPET image collected with the 320 mm FOV scanner is far worse than that of the HQPET image scanned with uEXPLORER, cannot show clear texture details, and contains a substantial amount of noise, which affects the diagnosis results. Compared with LQPET, GAN-based CycleAGAN, CycleGAN, and Pix2Pix deep learning methods suppress image noise, significantly improve image quality, and maintain rich details and texture structures of PET images. However, the traditional method NLM makes all contours and textures in a predicted image extremely smooth, and BM3D overemphasizes contour information and ignores texture details. Hence, the effect of diagnosis is reduced. Compared with Pix2Pix and CycleGAN, CycleAGAN has better image quality and better texture matching with HQPET images. The image quality improvement effect of CycleAGAN is particularly obvious in the restoration of organ texture details, such as the location of the red box in the brain, lungs, and abdomen.

In quantitative analysis, CycleAGAN is compared with CycleGAN, Pix2Pix, NLM, and BM3D.  Table 2 shows the quantitative analysis results of the five methods in the three beds. The average NRMSE, PSNR, and SSIM between the predicted and real HQPET images obtained using CycleAGAN, CycleGAN, Pix2Pix, BM3D, and NLM methods are calculated. The proposed CycleAGAN achieves the best results in terms of NRMSE and SSIM in the three beds. The PSNR of BM3D reaches the highest value in all three beds. However, as shown in Figure 7, the contour information of the image predicted by BM3D is prominent, and thus, the detail texture is nearly completely lost. These results will affect the diagnosis effect of PET images.

#### 4.1.2. Radiologist Rating

With regard to the image quality scores provided by doctors, the distribution of the image quality scores for LQPET, HQPET, and estimated images from CycleAGAN, CycleGAN, Pix2Pix, BM3D, and NLM methods is shown in Figure 8. Figures 8(a)–8(c) show the scores of bed1, bed2, and bed3 respectively. Most of LQPET images scored 1 or 2, and only 7 cases in bed1 scored 3 or 4. The scores of HQPET images are mostly 4 or 5. Among 95 cases, only 3 and 4 of bed2 and bed3 are considered as low-quality images, respectively. The average scores of our proposed CycleAGAN are (4.11 ± 0.98, 4.10 ± 0.96, and 4.09 ± 0.94), respectively, and the score distribution is the closest to the ground-truth HQPET, far outperforming CycleGAN (average scores 3.72 ± 1.23, 3.68 ± 1.12, 3.70 ± 1.09), Pix2Pix (average scores 3.23 ± 1.02, 3.25 ± 1.03, 3.20 ± 1.05), NLM (average scores 1.82 ± 0.70, 1.81 ± 0.68, 1.78 ± 0.68), and BM3D (average scores 2.49 ± 0.87, 2.51 ± 0.92, 2.50 ± 0.95).

### 4.2. Result of Generalization Experiments

In this section, we test the generalization ability of the model in five additional cases. The uEXPLORER is used to collect the raw data of five additional cases and reconstruct them into three discontinuous LQPET–HQPET image pairs. The FOV of each bed position is 250 mm, and the bed positions correspond to the head (bed1), lung (bed2), and abdomen (bed3). The reconstruction parameters are the same as those of the 320 mm scanner. The corresponding slices of each bed position are 179 in the head, 125 in the lung, and 125 in the abdomen. The data of the five cases are input into the trained model as a validation set to test the generalization performance of the model.

Qualitative and quantitative analysis results are shown in Figure 9 and Table 3, respectively. Each row in Figure 9 shows the enhancement effect of each bed in different methods. In the comparison between Figures 7 and 9, the overall image quality in Figure 9 is not as good as that in Figure 7. In the first two columns of Figure 9, the LQPET image collected in five minutes with the 250 mm FOV scanner is far from the visual effect of clinical diagnosis, whereas the HQPET image scanned by uEXPLORER shows clear texture details. The red box in Figure 9 shows the texture detail recovery ability of each method. The result of CycleAGAN is the closest to that of HQPET, and other methods cannot restore the most valuable texture information in the LQPET image with a substantial amount of noise.

A considerable amount of noise is found in the LQPET image collected with the 250 mm scanner, and the quantitative analysis results in Tables 2 and 3 show that all the values in Table 3 are slightly lower than those in Table 2. All the methods can effectively enhance LQPET image quality. The proposed CycleAGAN achieves the best results in terms of the NRMSE and SSIM values of each bed and the maximum PSNR value of bed1. In this experiment, although CycleGAN achieves the maximum PSNR values of bed2 and bed3, the image quality is second only to that of CycleAGAN. According to the results in Tables 2 and 3, the proposed method is less affected by the accuracy of the scanner in a certain range and can achieve good results. Therefore, the proposed image quality improvement method CycleAGAN has great generalization ability.

## 5. Discussion

The purpose of most existing image quality enhancement algorithm [24, 27, 28, 43] is to reduce the radiation of a radioactive tracer in the human body and ensure image quality while reducing the dose. The common problem of these algorithms [24, 27, 28, 43] is that they ignore the impact of hardware device on image quality [44], and they cannot be integrated with conventional short-axis PET scanner. In this paper, our method improves the image quality collected by different FOVs and effectively improves the structural consistency of the synthesized images with HQPET. Another challenge of PET image generation is the construction of texture details. Given that a large amount of noises mix with texture features in low-quality images, the method of Zhao and Zhou [27, 28] inevitably treats some fine textures as noise despite resulting in good image quality; nevertheless, these fine textures can provide useful clinical information for the diagnosis, although they present a huge challenge to PET image reconstruction. We have incorporated the attention mechanism into the CycleGAN generator network to generate HQPET images with low noise and clear texture. In addition, owing to the insufficient amount of data, current methods randomly divide image patches and generate complete image outputs by overlapping patch blocks. Although these methods expand the amount of data and save computing resources, the global features of the images cannot be collected, and the collected neighborhood information is insufficient. The sample size of the dataset used in our work can well meet the number of samples required for deep learning, and inputting the entire image into the network during training can extract more global and texture features.

Although the model proposed in this paper achieves convincing results, some limitations remain. Our method can improve the quality of LQPET collected with different FOV, but it still cannot completely overcome the differences between different scanners. Compared with other GAN and CNN-based methods, CycleAGAN needs a longer training time and more computing resources. Future work should consider a more efficient network architecture. In addition, data sets are greatly limited, and the pairing of HQPET and LQPET in space is required. Although the same patient undergoes two consecutive examinations, differences in space and radiation attenuation are still found. Moreover, although the brain, lungs, and abdomen are trained separately and achieved considerable results, the discontinuity between each bed is found, which may lead to some bad results in practical application. Nevertheless, these proposed problems provide directions for future work.

## 6. Conclusion and Future Work

In summary, a deep learning CycleAGAN method with the attention mechanism and supervised loss was proposed to improve the image quality of the short-axis PET scanner. The effectiveness of the model is verified using the data of 386 cases collected with a total-body PET scanner. The proposed method aims to (1) obtain a high-quality reconstruction image with low noise and clear texture with the CycleAGAN method, (2) use the attention mechanism to shift the focus to the representative features of space and channel in the reconstruction of fine texture information, (3) use paired data corresponding to spatial position for training, add supervised loss, and reduce the influence of deformation on generated images. The experimental results show that the method not only can improve the image quality of a PET scanner with 320 mm FOV but also achieves good results on a scanner with 250 mm FOV. Patients and radiologists can benefit from the CAD system [45] integrated with the CycleAGAN method, which plays a significant role in image diagnosis.

In future work, the proposed method may be applied to scanners with different FOV and all parts of the body to prove the wide adaptability of this method. We will expand the scope of its application by using it to improve the quality of images obtained with other medical image scanners.

## Figures and Tables

**Figure 1:** Comparison of the image quality between a short-axis and total-body PET scanners. (a, d) Brain PET images. (b, e) Lung PET images. (c, f) Abdomen PET images. The images scanned by the short-axis scanner are shown in the first row, and the images scanned by the total-body scanner are shown in the second row.

**Figure 2:** CycleAGAN framework. Overview of the proposed framework for LQPET image quality improvement.

**Figure 3:** The overview of CBAM. The module has two sequential submodules: channel and spatial.

**Figure 4:** The architecture of each attention submodule. The channel attention module uses both max-pooling outputs and average-pooling outputs with a common convolutional network; the spatial attention module uses two combined outputs converged along the channel axis and forwards them to a convolution layer.

**Figure 5:** Generator. A generator architecture in the proposed framework.

**Figure 6:** Discriminator. A discriminator architecture in the proposed framework.

**Figure 7:** Simple images of LQPET (320 mm), HQPET (1940 mm), and estimated PET images from CycleAGAN, CycleGAN, Pix2Pix, NLM, and BM3D methods. (a) Brain PET images. (b) Lung PET images. (c) Abdomen PET images. Rows 1, 2, and 3 in each subgraph are PET images in the axial, coronal, and sagittal direction, respectively.

**Figure 8:** Image quality score given by two radiologists. (a–c) The scores of bed1, bed2, and bed3, respectively. At the top of each bar are the mean scores and standard deviations.

**Figure 9:** Simple images of LQPET (250 mm), HQPET (1940 mm), and estimated PET images from CycleAGAN, CycleGAN, Pix2Pix, NLM, and BM3D methods. Row 1 presents brain PET images. Row 2 displays lung PET images. Row 3 shows abdomen PET images.

**Table 1:** Evaluation scale of radiologist experts.

Evaluation scale	Score
The image is not diagnostic, too large noise, poor lesions	1
Image quality is acceptable, large noise, poor description of lesions, reduce diagnostic confidence	2
Image quality is acceptable, reaching the clinical routine image quality	3
Image quality is better than average image quality	4
Image quality is excellent, low noise, the lesion is clear, no artifact	5

**Table 2:** Quantitative comparison on LQPET images from the scanner with 320 mm FOV.

Data	Methods	NRMSE	PSNR (dB)	SSIM
bed1	LQPET	0.248 ± 0.20	31.595 ± 4.67	0.915 ± 0.08
	**CycleAGAN**	**0.219** ± **0.09**	34.003 ± 2.11	**0.950** ± **0.03**
	CycleGAN	0.340 ± 0.19	31.263 ± 3.70	0.900 ± 0.07
	Pix2Pix	0.292 ± 0.16	33.171 ± 4.49	0.931 ± 0.05
	NLM	0.303 ± 0.24	34.309 ± 3.85	0.883 ± 0.06
	BM3D	0.244 ± 0.13	**34.525** ± **3.67**	0.883 ± 0.06

bed2	LQPET	0.258 ± 0.14	30.293 ± 5.28	0.910 ± 0.05
	**CycleAGAN**	**0.222** ± **0.06**	30.228 ± 2.79	**0.927** ± **0.02**
	CycleGAN	0.241 ± 0.09	31.284 ± 5.05	0.921 ± 0.03
	Pix2Pix	0.241 ± 0.11	30.685 ± 3.63	0.918 ± 0.03
	NLM	0.258 ± 0.14	31.454 ± 4.92	0.898 ± 0.03
	BM3D	0.241 ± 0.10	**31.972** ± **5.35**	0.912 ± 0.05

bed3	LQPET	0.263 ± 0.14	34.973 ± 8.13	0.948 ± 0.05
	**CycleAGAN**	**0.257** ± **0.07**	36.065 ± 6.87	**0.958** ± **0.02**
	CycleGAN	0.271 ± 0.14	36.286 ± 6.91	0.952 ± 0.03
	Pix2Pix	0.273 ± 0.12	35.526 ± 8.30	0.949 ± 0.04
	NLM	0.276 ± 0.14	35.319 ± 5.24	0.937 ± 0.04
	BM3D	0.300 ± 0.17	**36.315** ± **7.27**	0.934 ± 0.04

Best results and methods are highlighted.

**Table 3:** Quantitative comparison of LQPET images from the scanner with 250 mm FOV.

Data	Methods	NRMSE	PSNR (dB)	SSIM
bed1	LQPET	0.257 ± 0.23	30.444 ± 4.22	0.886 ± 0.09
	**CycleAGAN**	**0.225** ± **0.12**	**31.975** ± **2.76**	**0.927** ± **0.04**
	CycleGAN	0.332 ± 0.21	28.726 ± 2.78	0.885 ± 0.05
	Pix2Pix	0.349 ± 0.29	29.387 ± 2.82	0.892 ± 0.04
	NLM	0.305 ± 0.29	31.063 ± 2.88	0.837 ± 0.06
	BM3D	0.242 ± 0.13	31.160 ± 3.07	0.862 ± 0.04

bed2	LQPET	0.268 ± 0.20	29.602 ± 4.27	0.874 ± 0.05
	**CycleAGAN**	**0.205** ± **0.09**	29.920 ± 2.87	**0.919** ± **0.03**
	CycleGAN	0.218 ± 0.10	**30.919** ± **3.09**	0.908 ± 0.03
	Pix2Pix	0.207 ± 0.08	30.119 ± 2.81	0.906 ± 0.03
	NLM	0.273 ± 0.21	29.708 ± 4.11	0.861 ± 0.04
	BM3D	0.211 ± 0.10	30.106 ± 4.36	0.875 ± 0.05

bed3	LQPET	0.278 ± 0.13	33.240 ± 5.40	0.899 ± 0.06
	**CycleAGAN**	**0.258** ± **0.10**	33.892 ± 4.67	**0.933** ± **0.03**
	CycleGAN	0.265 ± 0.10	**34.365** ± **5.41**	0.924 ± 0.03
	Pix2Pix	0.276 ± 0.10	32.422 ± 6.19	0.920 ± 0.04
	NLM	0.271 ± 0.14	33.872 ± 4.86	0.896 ± 0.04
	BM3D	0.256 ± 0.11	34.154 ± 4.63	0.910 ± 0.03

Best results and methods are highlighted.

## Data Availability

The data used to support the findings of this study may be released upon application to the Henan Provincial People's Hospital, which can be contacted at ypwu@ha.edu.cn.
